The article "Association of Polymorphism rs198977 in Human Kallikrein-2 Gene (KLK2) with Susceptibility of Prostate Cancer: A Meta-Analysis" was retracted in 2016. Reasons: compromised peer review; false authorship; ethical violations by an author.

# Association of Polymorphism rs198977 in Human Kallikrein-2 Gene (KLK2) with Susceptibility of Prostate Cancer: A Meta-Analysis

**DOI:** 10.1371/journal.pone.0065651

**Published:** 2013-06-18

**Authors:** Lishan Wang

**Affiliations:** 1 Bio-X Institutes, Key Laboratory for the Genetics of Developmental and Neuropsychiatric Disorders (Ministry of Education), Shanghai Jiao Tong University, Shanghai, P.R. China; 2 FengHe (ShangHai) Information Technology Co., Ltd, Shanghai, P.R. China; IPO, Inst Port Oncology, Portugal

## Abstract

**Objectives:**

To assess the association of polymorphism rs198977 in the human kallikrein-2 gene (KLK2) and risk of prostate cancer (PCa).

**Methods:**

Two investigators independently searched the PubMed, Elsevier, EMBASE, Web of Science, Wiley Online Library and Chinese National Knowledge Infrastructure (CNKI). Pooled odds ratios (ORs) and 95% confidence intervals (95% CIs) for rs198977 and PCa were calculated in a fixed-effects model (the Mantel-Haenszel method) and a random-effects model (the DerSimonian and Laird method) when appropriate.

**Results:**

Six studies met the inclusion criteria in this meta-analysis, which included 5859 PCa cases and 4867 controls. Overall, rs198977 was associated with the PCa risk (TT+CT vs. CC, pooled OR = 1.163, 95% CI = 1.076–1.258, P-value <0.0001). When stratified by ethnicity, significant association was observed in Caucasian samples under both allele comparison (T vs. C, pooled OR = 1.152, 95% CI = 1.079–1.229, P-value <0.0001) and dominant model (TT+CT vs. CC, pooled OR = 1.197, 95% CI = 1.104–1.297, P-value <0.0001). In the overall analysis, a comparably significant increase in the frequency of allele T for rs198977 was detected between cases and controls in Caucasian.

**Conclusion:**

This meta-analysis suggests that rs198977 of KLK2 was associated with susceptibility of PCa in Caucasian and the allele T might increase the risk of PCa in Caucasian.

## Introduction

Prostate cancer (PCa) is the most commonly diagnosed visceral malignancy accounting for more than one-third of all incident cancers and is the second-leading cause of cancer deaths in men in the United States and the western world [1] [2]. Prostate-specific antigen (PSA) has been used for detecting PCa since 1994 [3]. The wide availability of total PSA revolutionized PCa screening and ushered in the PSA era resulting in a decrease of PCa metastasis and death. Several novel blood-based biomarkers, such as human glandular kallikrein 2 (hK2) may also help PCa diagnosis, staging, prognostication, and monitoring [4].

There is considerable evidence for a genetic basis underlying risks for PCa [5], and it is among the most heritable of the common cancers with a heritability of 42% estimated from a twin study [6].The kallikrein (KLK) gene family, consisting of 15 genes spanning a region of approximately 300 kb on 19q13.4, encodes the largest known cluster of serine-proteases in the human genome [7] [8]. Two of the classical KLK genes, KLK3 and KLK2, that are contiguously located, are expressed almost exclusively in prostate tissue. KLK3 encodes PSA [9], which is produced primarily by prostate epithelium and is widely used as a tumor marker for early detection and monitoring of PCa [10] [11]. KLK2 encodes hK2 that is specific for the prostate and regulates the expression of PSA [12]. They share an 80% sequence homology and are both primarily expressed in the prostate gland [13]. Using a set of single nucleotide polymorphisms (SNPs) that span the KLK2 region, Nam *et al.* have demonstrated that KLK2 variants correlate with hK2 serum levels [14]. In addition, Stenman *et al.* showed that hK2 mRNA expression was significantly higher in PCa tissue compared with benign tissue [15]. Moreover, hK2 is expressed at higher level in poorly differentiated cancers and is a likely candidate for prostate carcinogenesis [16].

All of these observations strongly implicate KLK2 as a plausible candidate gene involved in PCa susceptibility. During this decade, a number of studies have assessed the association between polymorphism rs198977 in KLK2 and risk of PCa in different populations; however, the results are inconsistent and inconclusive [17] [18]. Different methodologies have been used, and in particular, samples are collected from all over the world. Therefore, it is not surprising that there has been a lack of replication in different studies. By using all the available published data to increase the statistical power, it was hypothesized that a meta-analysis might allow plausible candidate genes to be excluded and causative genes to be identified with reliability. To confirm whether the polymorphism rs198977 in KLK2 is associated with susceptibility of PCa, we have taken a meta-analysis in which all the published case-control studies are processed.

## Materials and Methods

### Literature Search

Published reports assessing the association between polymorphism of KLK2 and risk of PCa were collected through a comprehensive search of six databases, including PubMed, Elsevier, EMBASE, Web of Science, Wiley Online Library and Chinese National Knowledge Infrastructure (CNKI). The search terms were as follows: (‘KLK2’ OR ‘kallikrein-2’ OR ‘hK2’) AND (‘prostate cancer’). Searching was completed on Nov 1, 2012. Publication date and publication language were not restricted in our search. Meanwhile, reference lists were examined manually to further identify potentially relevant studies. Unpublished reports were not considered. If more than one article was published by the same author using the same case series, the one investigating the most individuals was selected.

### Inclusion and Exclusion Criteria

Abstracts of all citations and retrieved studies were reviewed. Studies meeting the following criteria were included: (1) Using a case–control design; (2) Detecting the relationship between the polymorphism rs198977 and PCa; (3) Providing available genotype data of rs198977. Studies were excluded if one of the following existed: (1) The design was based on family or sibling pairs; (2) The genotype frequency of rs198977 was not reported; (3) The association of rs198977 with susceptibility of PCa (e.g. cancer progression and mortality) was not detected, or (4) There was insufficient information for extraction of data.

### Data Extraction

All data were extracted independently by two reviewers (lishan wang and weidong zang) according to the inclusion criteria listed above. The results were compared and disagreements were discussed and resolved with consensus. Evaluation was based on title and abstract whenever available. Full text articles of potentially relevant studies were obtained and re-evaluated for inclusion. The following characteristics were collected from each study using an Excel data extraction form: first author, year of publication, country of sample, ethnicity, numbers of cases and controls, main background of samples, and genotyping methods (Table 1).

**Table 1:** Characteristics of studies included in the meta-analysis.

Author	Year	Country	Ethnicity	No.(cases/controls)	Matching criteria	Genotyping methods	Ref.
Nam, R. K.	2003	Canada	Caucasian	616/671	Age, race	PCR-RFLP	[17]
Chiang,C.H	2005	China	Asian	254/168	Age, race	PCR-RFLP	[18]
Nam, R. K.	2005	Canada	Caucasian	996/1092	Age, race	PCR-RFLP	[19]
Mittal,R. D.	2007	India	Asian	135/142	Age, race	PCR-RFLP	[20]
Ahn, J.	2008	USA	Caucasian	1172/1157	Age, race	Sequencing	[21]
Klein,R.J.(a)*	2010	Sweden	Caucasian	1397/724	Age, race	Sequencing	[22]
Klein,R.J.(b)*	2010	Sweden	Caucasian	1219/842	Age, race	Sequencing	[22]

* Klein’s study included two separate groups of samples, data was extracted according to the groups (a and b) as they were independent with each other and analyzed respectively in the initial study. PCR-RFLP: Polymerase chain reaction-restriction fragment length polymorphism.

### Statistical Analysis

The statistical analysis was conducted using STATA 11.0 (Stata Corp LP, College Station, TX, United States); P-value <0.05 was considered statistically significant. Hardy-Weinberg equilibrium (HWE) in the controls was tested by the chi-square test for goodness of fit, and a P –value <0.05 was considered as significant disequilibrium. Pooled odds ratio (ORs) were calculated for allele comparison (T vs. C), dominant model (TT+CT vs. CC), and recessive model (TT vs. CC+CT), respectively. The significance of pooled ORs was determined by Z-test and P-value <0.05 was considered as statistically significant.

The OR and 95% CI were estimated for each study in a random-effects model or in a fixed-effects model. Heterogeneity among studies was examined with the χ^2^ -based Q testing and *I^2^* statistics [19]. P-value <0.1 was considered significant for the χ^2^-based Q testing and I^2^ was interpreted as the proportion of total variation contributed by between-study variation. If there was a significant heterogeneity (P-value <0.1), we selected a random-effects model (the DerSimonian and Laird method) to pool the data. If not, we selected a fixed-effects model (the Mantel-Haenszel method) to pool the data. Heterogeneity was also quantified using the *I^2^* metric (*I^2^*<25%, no heterogeneity; *I^2^* = 25–50%, moderate heterogeneity; *I^2^*>50%, large or extreme heterogeneity) [25]. Publication bias was examined with funnel plots and with the Egger’s tests [20] [21]. If there is evidence of publication bias, the funnel plot is noticeably asymmetric. For the Egger’s tests the significance level was set at 0.05.

## Results

### Study Characteristics

A total of 121 papers were retrieved after the first search, and 115 of these were excluded from the analysis for reasons detailed in Figure 1. Only 6 case-control studies met the inclusion criteria in this meta-analysis, which included 5859 PCa cases and 4867 controls [17] [18]. Characteristics of studies included in the meta-analysis were presented in Tables 1 and 2. The qualities of the studies were considered acceptable for our meta-analysis. We calculated HWE for all six publications and found that only Klein’s study [18] was inconsistent with Hardy-Weinberg disequilibrium (P-value = 0.01). The flow chart of selection of studies and reasons for exclusion was presented in Figure 1. Studies had been carried out in Canada (n = 2), Sweden (n = 1), USA (n = 1), China (n = 1) and India (n = 1). Four studies [17][22] [23] used Caucasian samples while two studies [24][25] used Asian samples.

**Figure 1:** Flow chart of selection of studies and specific reasons for exclusion from the meta-analysis.

**Table 2:** Genotype frequencies of rs198977 in studies included in the meta-analysis.

Author	Year	Case genotype^a^			Control genotype^b^			HWE^c^	Ref.
		CC	CT	TT	CC	CT	TT		
Nam, R. K.	2003	315	251	50	394	240	37	0.873	[17]
Chiang,C.H	2005	169	83	2	94	52	9	0.195	[18]
Nam, R. K.	2005	522	394	80	621	413	58	0.782	[19]
Mittal,R. D.	2007	78	50	7	72	52	18	0.211	[20]
Ahn, J.	2008	621	469	82	660	428	69	0.719	[21]
Klein,R.J.(a)	2010	788	515	94	443	233	48	0.052	[22]
Klein,R.J.(b)	2010	670	460	89	483	287	72	0.010	[22]

a Absolute number of patients;

b Absolute number of controls;

c HWE: Hardy-Weinberg equilibrium, it was evaluated using the goodness-of-fit chi-square test. P-values were presented. P<0.05 was considered representative of a departure from HWE.

### Evaluation of rs198977 and Association with PCa

There were six case-control studies [17] [18]which had been performed to study the polymorphism rs198977 and PCa risk. Results of the meta-analysis were shown in Table 3. Overall, when all the eligible studies were pooled into the meta-analysis, we found that a significant PCa risk was associated with rs198977 polymorphism in a dominant model (TT+CT vs. CC, pooled OR = 1.163, 95% CI = 1.076–1.258, P-value <0.0001); while no significant association was observed in either allele comparison (T vs. C, pooled OR = 1.077, 95% CI = 0.957–1.212, P-value = 0.216) or recessive model (TT vs. CT+CC, pooled OR = 0.993, 95% CI = 0.718–1.373, P-value = 0.964).

**Table 3:** Pooled odds ratio for rs198977 in meta-analyses.

Population	Genetic Model	Pooled OR(95% CI)	P-value^a^	P-value^b^ (Publication bias)	P-value^c^ (heterogeneity)	I^2^
All	Allele T vs.C	1.077(0.957–1.212)	0.216	0.047	0.006	67.0%
	Dominant	1.163(1.076–1.258)	<0.0001	0.050	0.143	37.4%
	Recessive	0.993(0.718–1.373)	0.964	0.093	0.001	72.2%
Caucasian	Allele T vs.C	1.152(1.079–1.229)	<0.0001	0.328	0.319	14.9%
	Dominant	1.197(1.104–1.297)	<0.0001	0.129	0.703	0.0%
	Recessive	1.173(0.930–1.480)	0.177	0.328	0.077	52.5%
Asian	Allele T vs.C	0.701(0.542–0.906)	0.007	–	0.928	0.0%
	Dominant	0.765(0.560–1.045)	0.092	–	0.924	0.0%
	Recessive	0.278(0.128–0.600)	0.001	–	0.239	27.8%

a Random-effects model was used when the p-value for heterogeneity test<0.10, otherwise the fixed-effect model was used.

b Egger’s test to evaluate publication bias, P –value <0.05 is considered statistically significant.

c P-value <0.1 is considered statistically significant for Q statistics.

When studies were stratified by ethnicity, significant associations were observed in Caucasian group in both allele comparison (T vs. C, pooled OR = 1.152, 95% CI = 1.079–1.229, P-value <0.0001) and dominant model (TT+CT vs. CC, pooled OR = 1.197, 95% CI = 1.104–1.297, P-value <0.0001) (Figure 2); while no significant association was observed in Caucasian group in recessive model (TT vs. CT+CC, pooled OR = 1.173, 95% CI = 0.930–1.480, P-value = 0.177). In addition, significant associations were observed in Asian group in both allele comparison (T vs. C, pooled OR = 0.701, 95% CI = 0.542–0.906, P-value = 0.007) and recessive model (TT vs. CT+CC, pooled OR = 0.278, 95% CI = 0.128–0.600, P-value = 0.001); while no significant association was observed in Asian group in dominant model (TT+CT vs. CC, pooled OR = 0.765, 95% CI = 0.560–1.045, P-value = 0.092).

**Figure 2:** Forest plots of studies with Caucasian samples under dominant model (a) and Allele comparison model (b).

### Sensitivity Analysis

The influence of a single study on the overall meta-analysis was investigated by omitting one study at a time, and the omission of any study made no significant difference, indicating that our results were statistically reliable.

### Evaluation of Heterogeneity

For all samples, statistically significant heterogeneity was observed under both allele comparison (T vs. C, P-value by χ^2^ -based Q testing = 0.006 and *I^2^* = 67.0%) and recessive model (TT vs. CT+CC, P-value by χ^2^ -based Q testing = 0.001 and *I^2^* = 72.2%), but no significant heterogeneity was observed under dominant model (TT+CT vs. CC, P-value by χ^2^ -based Q testing = 0.143 and *I^2^* = 37.4%). Then subgroup analysis was carried out. When studies were stratified by ethnicity, no statistically significant heterogeneity was observed in Caucasian under either allele comparison (T vs. C, P-value by χ^2^ -based Q testing = 0.319 and *I^2^* = 14.9%) or dominant model (TT+CT vs. CC, P-value by χ^2^ -based Q testing = 0.703 and *I^2^* = 0.0%), but there was significant heterogeneity under recessive model (TT vs. CT+CC, P-value by χ^2^ -based Q testing = 0.077 and *I^2^* = 52.5%). For Asian, no statistically significant heterogeneity was observed under any model (all P-values by χ^2^ -based Q testing >0.1 and *I^2^*<50%). Results of heterogeneity were shown in Table 3.

### Publication Bias

Funnel plot and Egger’s test were performed to assess the publication bias of the literature. Results publication bias was shown in Table 3. For all samples, publication bias was observed under allele comparison (T vs. C, P-value of Egger’s test = 0.047). After samples were stratified by ethnicity, no publication bias was observed under any model (all P-value of Egger’s test >0.05). Symmetrical funnel plots were obtained for Caucasian (Figure 3), but Funnel plot and Egger’s test were not available for Asian samples because of the small sample size.

**Figure 3:** Funnel plots of studies with Caucasian samples under dominant model (a) and Allele comparison model (b).

## Discussion

The data from this meta-analysis showed a significant increase in frequency of genotype TT+CT of rs198977 polymorphism in patients with PCa than controls, which suggested that genotype TT+CT might increase the risk of PCa with pooled OR of 1.163. When stratified the samples by their ethnicity, the frequencies of both the allele T and genotype TT+CT in Caucasian had significant increase in cases than controls with pooled OR of 1.152 and 1.197, respectively; but things became different for Asian, there was a significant decrease in frequency of allele T in cases than control with pooled OR of 0.701. Though results from Asian samples indicated allele C of rs198977 was the risk factor, it still be under discussion because of the small sample size in our analysis. But the results clearly suggested that allele T of rs198977 was a moderate risk factor of PCa for Caucasian. In addition, Mikolajczyk *et al.* showed that increased hK2 expression in PCa tissues could influence cancer biology not only by activating uPA but also by inactivating its primary inhibitor, plasminogen activator inhibitor [26]. And results from transgenic mice demonstrate, with biologically relevant models, that KLK2 is the protease responsible for activating PSA [27]. Variants on KLK2 gene may affect the expression of hK2, and thus its biological function might be altered. These previous findings support our results and give us possible explanation to the mechanism.

The degree of heterogeneity is one of the major concerns in meta-analysis as non-homogeneous data are liable to result in misleading results. In the present study, the *Q* testing and *I*^2^ statistics were carried out to test the significance of heterogeneity. For all samples, significant heterogeneity existed under allele comparison and recessive model. After stratifying the samples according to their ethnicity, the heterogeneity decreased. For Caucasian samples, significant heterogeneity was observed under recessive model, while no statistically significant heterogeneity was observed under any model in Asian samples. The results indicated ethnicity might play an important role in genetic heterogeneity of rs198977. In other words, there exist heterogeneity of rs198977 between Caucasian and Asian according to our results.

Publication bias is another important factor affecting the quality of meta-analysis. In order to assess publication bias, funnel plot and Egger’s test were performed. Publication bias was observed under allele comparison when all studies were included. After removing Asian samples, no publication bias was observed under any model and symmetrical funnel plots were obtained for Caucasian (all P-value of Egger’s test >0.05) (Table 3 and Figure 3). This indicated that two studies with Asian samples might be responsible for the publication bias, but the reason could not be exactly determined as Funnel plot and Egger’s test were not available for only two studies. Moreover, we performed a sensitivity analysis by removing one study each time and re-running the model to determine the effect on each overall estimate. The estimates changed little, which implied that our results were statistically reliable.

However, there are still some limitations in this meta-analysis. (1) In six studies included for our analysis, two of them are Asian samples occupied only 6.52% of whole samples, so such results should be interpreted with caution; (2) Because the samples from 5 countries and controls were not uniform, as in most meta-analyses, results should be interpreted with caution; and (3) meta-analysis is retrospective research that is subject to methodological limitations. In order to minimize the bias, we used explicit methods for study selection, data extraction and data analysis. Nevertheless, our results should be interpreted with caution.

This meta-analysis suggests that the polymorphism rs198977 of KLK2 was associated with susceptibility of prostate cancer in Caucasian and the allele T might increase the risk of prostate cancer. The pooled ORs in this study suggest that allele T and genotype TT+CT both have modest but definite genetic effect on prostate cancer in Caucasian. Larger and well-designed studies based on different ethnic groups are needed to confirm our results, especially for Asian samples.

## Supporting Information

Checklist S1 **PRISMA checklist**.
(DOC)
